# Multitask Interactive Attention Learning Model Based on Hand Images for Assisting Chinese Medicine in Predicting Myocardial Infarction

**DOI:** 10.1155/2021/6046184

**Published:** 2021-10-26

**Authors:** Qida Wang, Chenqi Zhao, Yan Qiang, Zijuan Zhao, Kai Song, Shichao Luo

**Affiliations:** College of Information and Computer, Taiyuan University of Technology, Taiyuan, China

## Abstract

Acute myocardial infarction (AMI) is one of the most serious and dangerous cardiovascular diseases. In recent years, the number of patients around the world has been increasing significantly, among which people under the age of 45 have become the high-risk group for sudden death of AMI. AMI occurs quickly and does not show obvious symptoms before onset. In addition, postonset clinical testing is also a complex and invasive test, which may cause some postoperative complications. Therefore, it is necessary to propose a noninvasive and convenient auxiliary diagnostic method. In traditional Chinese medicine (TCM), it is an effective auxiliary diagnostic strategy to complete the disease diagnosis through some body surface features. It is helpful to observe whether the palmar thenar undergoes hypertrophy and whether the metacarpophalangeal joint is swelling in detecting acute myocardial infarction. Combined with deep learning, we propose a depth model based on traditional palm image (MTIALM), which can help doctors of traditional Chinese medicine to predict myocardial infarction. By building the shared network, the model learns information that covers all the tasks. In addition, task-specific attention branch networks are built to simultaneously detect the symptoms of different parts of the palm. The information interaction module (IIM) is proposed to further integrate the information between task branches to ensure that the model learns as many features as possible. Experimental results show that the accuracy of our model in the detection of metacarpophalangeal joints and palmar thenar is 83.16% and 84.15%, respectively, which are significantly improved compared with the traditional classification methods.

## 1. Introduction

Acute myocardial infarction (AMI) is the myocardial necrosis caused by acute and persistent ischemia and hypoxia of the coronary artery. It is the most serious and dangerous disease among cardiovascular diseases. In recent years, the number of patients has shown an obvious upward trend, among which the elites under the age of 45 in various industries have become the high-risk population prone to sudden death of myocardial infarction due to work pressure, overtime, and staying up late and other reasons. Therefore, how to timely detect and diagnose the disease before the onset and remind patients of prevention and maintenance is a major problem in the field of medicine at present. However, there are still some problems in clinical detection and diagnosis: first, the symptoms of patients with myocardial infarction before onset are not obvious, although patients will have chest pain and stuffy symptoms before the onset of the disease; these symptoms are not typical clinical symptoms, and patients often take it lightly. Second, there is no test for myocardial infarction in the routine physical examination. Although coronary angiography is the “gold standard” for the diagnosis of myocardial infarction, this method still is expensive, complex and cumbersome, and invasive. It will not only cause some harm to patients but also cause some postoperative complications. As a result of the above problems, the onset of myocardial infarction cannot be treated in time, leading to a high mortality rate.

Considering these problems with using traditional medical techniques to diagnose AMI, it is necessary to develop a noninvasive and convenient auxiliary diagnostic system to detect and prevent this disease. Recently, many researchers have attempted to implement and apply noninvasive methods based on the combination of computerized analysis and traditional Chinese medicine [1–4]. In many works [5–15], emphasis has been placed on disease diagnosis based on body surface features, which confirms the superiority and rationality of noninvasive methods. Wang et al. [16] designed a novel device to accurately capture tongue and face images for diagnostic purposes. In addition, a new tongue color space is proposed, which can represent tongue images with 12 colors statistically. Their corresponding disease detection experiments demonstrated the effectiveness of these colors. In addition, Kim et al. [17] proposed a diagnostic system for heart disease by utilizing the color distribution around facial images. Similarly, another work based on facial images was used for hepatitis detection in [18] with an average accuracy of 73.6%. Yang et al. [6] also proposed a respiratory analysis system to diagnose diabetes based on acetone concentration. Although the above studies demonstrate the effectiveness of computer diagnosis in traditional Chinese medicine, to our knowledge, there are few or no studies on the application of hand images in the auxiliary diagnosis of (AMI). In the aspect of hand diagnosis in traditional Chinese medicine, because it takes into account the various body regions and characteristics that reflect the different states of our organs, when the human body has suffered or will suffer from some diseases, there will often be different shapes and colors on the specific parts of the patient's hand. For example, in people with heart disease, many have bruising and turning blue or even purple in the thenar area (the bulge of muscle under the thumb). Patients with insufficient blood supply to the heart muscle will appear to have the metacarpophalangeal joint swelling phenomenon. Traditional Chinese medicine doctors can make an accurate judgment on whether patients are at risk of myocardial infarction by observing various features of the hand or face. Therefore, many patients with AMI are more inclined to be initially diagnosed by traditional Chinese medicine doctors through inspection. However, hand diagnosis in traditional Chinese medicine requires diagnostic physicians to have many years of medical experience. Different physicians have slightly different standards for hand diagnosis. As a result, the number of doctors is small, but the number of patients is large, the waiting time of patients is long, and doctors are under great pressure for diagnosis. With the rapid development of deep learning technology, how to combine traditional Chinese medicine hand diagnosis with artificial intelligence technology has become an important issue.

However, in the prediction and diagnosis of AMI by deep learning, more work focuses on the auxiliary prediction and diagnosis of myocardial infarction based on electrocardiogram (ECG) data and Magnetic Resonance Imaging (MRI) data. To our knowledge, there are no studies on the diagnosis of myocardial infarction (MI) based on traditional images. Baloglu et al. [19] achieved good results in the diagnosis of AMI by constructing an end-to-end deep learning model based on standard 12-lead ECG signals. Wei et al. [20] used Tunable Quality Factor (Q-Factor) Wavelet (TQWT) for Variational Mode Decomposition (VMD). The representative features were extracted by phase space reconstruction (PSR) and other methods, and then, the neural network modeling was used for myocardial infarction detection. Many recent studies [21–23] have achieved certain results in the diagnosis of myocardial infarction by using electrocardiogram data combined with a deep learning algorithm. But these studies use medical data (ECG, MRI, etc.) that are not readily available to the average person before they know they have a heart attack. But people will not obtain ECG, MRI, and other medical data without knowing that they have a heart attack.

To solve the above problems, we hope to establish a new depth model based on a traditional palm image, which can well assist traditional Chinese medicine in predicting myocardial infarction disease. The originality of our proposed approach has two main components. First of all, although many studies have attempted scientific work on the diagnosis of myocardial infarction, as far as we know, no work has attempted to study myocardial infarction through the combination of traditional Chinese medicine hand diagnosis and deep learning. Our work is a valuable attempt. In addition, our method can be combined with the professional hand diagnosis knowledge of TCM to simultaneously detect whether there are abnormal phenomena such as hypertrophy and swelling in two parts (metacarpophalangeal joints and palmar thenar) from the palm image, so as to further improve the detection efficiency. In conclusion, we propose a multitask interactive attentional learning model (MTIALM) to predict AMI based on hand images. Firstly, according to the hand images of AMI patients collected by the cooperative company and the disease labels marked by professional TCM physicians, we determined the optimal palm image size through experiments, which was used as the input of the whole model (Section 3.1). MTIALM is composed of a shared network and two task-specific attention branch networks (task M: detection of metacarpophalangeal joint swelling, task P: detection of palmar thenar hypertrophy). Shared network learning contains the characteristic information of all tasks (Section 3.2). For each task branch, soft attention is applied to learn task-specific features after extracting the output of different middle layers of the shared network, and finally, classification is made (Section 3.3). We propose a new module for information interaction (IIM) between tasks, which facilitates learning as much information as possible between different task branches (Section 3.4).

The contributions of this paper are as follows:

1. We propose a new method of deep learning based on a hand image to assist TCM diagnosis of AMI. A multitask interactive attention learning model (MTIALM) was designed to detect symptoms in two parts of the palm simultaneously to improve the diagnostic efficiency
2. A new information interaction (IIM) module is proposed to make the information exchange between different tasks better and make the model more targeted for training
3. The feasibility of this method is verified by experiments. The palm image is input into our proposed model, and the two tasks get their own classification results, respectively. The results obtained by our model have certain advantages compared with the current popular classification models

## 2. Related Work

### 2.1. Attention Mechanism

An attention mechanism automatically learns a group of weight coefficients through the network and emphasizes the regions we are interested in in the way of “dynamic weighting” and suppresses the irrelevant background regions at the same time. Inspired by the attention mechanism in machine translation, Xu et al. [24] published an article on the International Conference on Machine Learning (ICML) in 2015, which first applied the attention mechanism to the field of image description. It proposes two mechanisms of hard attention and soft attention at the same time and uses visualization technology to intuitively express the role of the attention mechanism. Hard attention is a random prediction that emphasizes dynamic change. Although it works well, its application is limited due to its nondifferentiable nature. On the contrary, soft attention is differentiable everywhere and can be obtained by neural network training based on a gradient descent method. Therefore, its application is relatively extensive. Hu et al. [25] model the interdependence between channels explicitly by building the “Squeeze-and-Excitation” block (SE block). Li et al. [26] were inspired by the concept block and SE block. From the perspective of multiscale features, they introduce multiple convolution kernel branches to learn the attention of feature graphs at different scales, so that the network can focus more on important scale features. In addition, He et al. [27] used the 1-dimensional sparse convolution operation to optimize the full-connection layer operations involved in the SE module, so as to significantly reduce the number of parameters and maintain a comparable performance. Through two-parallel channel attention and spatial attention, Park et al. [28] adopted expanded convolution to efficiently expand the receptive field and finally generated the final 3D attention MAP. Woo et al. [29] concatenated the two dimensions of channel and space and used global average pooling and maximum pooling to get the attention graph and then multiplied the attention graph with the input feature graph to refine the adaptive feature. Fu et al. [30] proposed a dual attention network that adaptively combines local features with global relevance and is used to solve the scene segmentation task. Cao et al. [31] proposed a lightweight global context modeling module that integrates spatial attention and channel attention into one module.

### 2.2. Multitask Learning

Since many problems in the real world cannot be decomposed into an independent subproblem, even if they can be decomposed, each subproblem is still related to each other and the rich correlation information among problems will be ignored in the process of decomposition. Therefore, multitasking learning is becoming more and more important. In the context of deep learning, a multitasking network has the potential to improve performance if the related tasks share complementary information or can act as a regulator for each other compared to the single-tasking situation. A lot of work [32–34] has demonstrated that multitasking networks can not only significantly reduce memory footprint and increase speed but also have the potential to improve performance between tasks. In hard parameter sharing, the parameter set is divided into shared and task-specific operations. In soft parameter sharing, each task is assigned its own set of parameters (i.e., task-specific networks) and feature sharing mechanisms handle the cross-task talk. UberNet [35] is the first multihead design architecture across different network layers and scales, handling low, medium, and advanced visual tasks in a unified architecture. Cross-stitch networks [36] use the linear combination activated in each layer of a specific task network as a means of soft feature fusion. By adopting the method of “single-tasking multiple tasks,” Maninis et al. [37] enabled the network to highlight the features suitable for the task through task-related feature adaptation or task attention. [38] considers the importance of task interaction from a multiscale perspective. Teichmann et al. [39] proposed a unified architecture for classification, detection, and semantic segmentation tasks and greatly increased the computational time from the perspective of real-time applications. [40] proposes a joint task recursive learning framework, which recursively refines the results of two t5asks through serialized task-level interactions and ultimately realizes a semantic segmentation and monocular depth estimation task. Multitask learning is currently a hot research field. The main idea is to learn multiple related tasks from a dataset at the same time. As an important research direction in multitask learning, an association rule mining (ARM) algorithm oriented to multitask has hardly been studied so far [41, 42]. The standard ARM algorithm discovers rules from the entire dataset instead of task-based, ignoring the relationship between tasks. [43] proposed the research of ARM based on multitask for the first time. It discovers rules by considering multiple tasks jointly. All the studies mentioned above have proven from different angles that multitask simultaneous learning can improve the learning ability of each individual task.

## 3. Materials and Methods

The overview of the proposed method is shown in Figure 1. We now introduce our proposed multitask-based attention learning framework model, which can be well applied to the hand-assisted diagnosis of AMI. Firstly, we preprocessed the collected palm image to obtain the region of interest (ROI) image and input it into the shared network to extract the common features (note that this shared network can be replaced with any popular classification network). Then, we designed a set of attention modules for different tasks, and these modules were combined with the common features extracted from the shared network to extract the specific features of specific tasks. In addition, we propose the information interaction module (IIM). It connects the specific features of different tasks in a new way and fuses the connected features to achieve further information interaction. We use a dimension reduction technique to reduce the feature channels such that the output features satisfy the channel dimension requirement of the next layers. We will further explain the three components of MTIALM in the following sections: the shared network, the task-specific attention branch, and the information interaction module.

### 3.1. Data Preprocessing

In this paper, in order to minimize the impact of environment, location, illumination, angle, and other factors, RGB images of the hands were collected with professional equipment. The device takes an image of a patient's hand at 1200 pixels by 1200 pixels, which is a higher resolution than normal images. However, for hand diagnosis of TCM, doctors of TCM seldom make diagnosis according to the finger region, and the main area of concern is the palm (the metacarpophalangeal joints, thenar, and other areas). Therefore, it is not beneficial for our work to directly input the original complete palm image as the model input. In addition, due to the high resolution of the original image, a deep neural network is needed for dimensionality reduction in order to predict our classification task. However, when too many convolutional layers are used in the network, a large number of parameters will be generated, which will lead to the problem of model overfitting. If we do not want to use too many convolutional layers, we need to use downsampling operations to reduce the size of the feature graph in order to meet the size requirements of the network. However, this would lose a lot of useful features, which would also be bad for our mission. In addition, a too large background area contains too much irrelevant information, which can cause the network to be unable to effectively focus on the key information contained in the ROI area. Therefore, we want the input of the model to include the part of the palm region as far as possible and avoid the interference of other regions (finger, wrist, background region, etc.), so as to learn the correct mapping relationship. Thus, we need to determine the optimal image size as an input to the overall model to ensure that we get as much useful information as possible.

At this point, we get an input image *X* ∈ *R*(*H*, *W*, *C*) with rich information, where *H* and *W* are the height and width of the patch image, respectively, and *C* is the number of channels of the patch image. In order to ensure that the palm area is located in the center of the image (patch), we labeled the area of interest in the image by referring to the professional diagnosis and treatment experience of a TCM doctor with 20 years of experience. In the natural unfolding state of the palm, as shown in Figure 2, the demarcation points between the middle finger and the palm were marked as *Y*_1_, the demarcation points between the palm and the wrist were marked as *Y*_2_, the demarcation points between the thumb and the palm were marked as *X*_1_, and the boundary on the other side of the palm was marked as *X*_2_. Then, Δ*X* and Δ*Y* (Δ*X*: 423 ± 16.26, Δ*Y*: 439 ± 27.15) are calculated as equation (1). Finally, as shown in equation (2), the larger one of the two values is selected to obtain *P*_size_. *P*_size_ is taken as the height and width of patch image size and is intercepted.

(1) $$\begin{array}{c} \left\{\begin{array}{c} \Delta X=\left|X_{1}-X_{2}\right|\\ \Delta Y=\left|Y_{1}-Y_{2}\right| \end{array}\right\}, \end{array}$$

(2) $$\begin{array}{c} P_{\text{size}}=\max\langle \Delta X,\Delta Y\rangle . \end{array}$$

As shown in Figure 3, in order to ensure that the entire palm region is included in the patch image, we counted the *P*_size_ corresponding to the palm region in all the palm images and finally found that the *P*_size_ of most samples was less than 460. Therefore, we decide to set the size of the patch image as 460 and feed it into the neural network as the input of the model.

### 3.2. Shared Network

The proposed multitask attention learning model (MTIALM) consists of three parts: the shared network for extracting common features, the attention network corresponding to each specific task, and the information interaction module (IIM) between tasks. The shared network can be switched according to specific tasks. After processing the data, we input it into the shared network for extracting common features. We use ResNet-18 as a shared network in our work. The deep residual network (ResNet) [44] has almost become the most widely used convolutional neural network (CNN) in the field of deep learning in recent years, and its main advantage is the shortcut structure constructed based on the residual learning concept. In the forward convolution, convolution of each layer actually only extracts part of the image information. As a result, the deeper the original image, the more serious the loss of information. However, if only a small part of the features in the original image is extracted, it is obvious that the phenomenon similar to underfitting will occur. Adding a shortcut structure is equivalent to adding all the information of the previous image in each block. In this way, more of the original information is preserved. When there is no shortcut, all samples are classified by using the most complex features, which is time-consuming and laborious. After adding a shortcut, it is equivalent to retaining some simple features for judgment, which not only accelerates the convergence of the network but also reduces the loss of information. For the proposed networks of different depths, such as ResNet-18, ResNet-34, and ResNet-50, we determined to use ResNet-18 as the shared network model after verification (Section 4.3).

In addition, we also applied transfer learning to extract common features by using the CNN model pretrained by ResNet-18 on the ImageNet [45] dataset. As far as we know, transfer learning requires that the source space and the target space are relatively similar. Because our hand images are also ordinary images rather than grayscale images or other medical images, we carried out network weight migration. This method can not only accelerate and optimize the learning efficiency of the model but also avoid the overfitting problem which may be caused by the small number of datasets.

### 3.3. Task-Specific Attention Branch Networks

We use common features extracted from different layers of the shared network to build task-specific attention modules. By cascading several attention modules together, a branching network of attention is formed and features related to a particular task are learned. As shown in Figure 1, the common features at different levels extracted from the shared network are represented as *f*(*i*), *i* = 1,2,3,4,5. Then, the output of the attention module is expressed as *f*_*m*_(*i*). It is worth noting that the first attention module of each branch only takes as input the shallowest common features extracted from the shared network. We divide each attention module into two parts, one of which is expressed as AMX-1 and the other as AMX-2 (*X* is the serial number of the notice module). In AMX-1, we conduct information fusion between the public features and the output of the attention module of the previous layer and carry out feature extraction through the convolutional layer. As shown in equation (3), we express the output of this stage as *f*′(*i*):

(3) $$\begin{array}{c} f^{\prime }\left(i\right)=\left\{\begin{array}{c} T\left(G\left(f\left(i\right)\right)\right),i=1\\ T\left(G\left(f\left(i\right)⊕f_{m}\left(i-1\right)\right)\right),i\geq 2 \end{array}\right\}, \end{array}$$

where ⊕ denotes the concatenation. *G* and *T* are convolutional layers with batch normalization [46]. Batch normalization is used to prevent overfitting of the model. *G* is composed of a [3 × 3] convolution kernel and activation function ReLU, and *T* is composed of a [1 × 1] convolution kernel and activation function sigmoid. We use a [1 × 1] convolution kernel in order to match the channel between the output feature of the previous layer of the attention module and the shared feature of this layer.

In order to better enable the network to learn the relevant characteristics of specific tasks, we set the second part AMX-2. In this part, we further exchange information between the output of the IIM block (Section 3.4) and the output of the previous part. As shown in equation (4), the output of AMX-2 in the second part is the output of the attention module *f*_*m*_(*i*):

(4) $$\begin{array}{c} f_{m}\left(i\right)=G\left(\left(f^{i}\left(i\right)+1\right)⊙f_{\text{IIM}}\left(i\right)\right),\;i=1. \end{array}$$

Here, *f*_IIM_(*i*) denotes the output of the IIM block for information interaction between branches. ⊙ denotes the element-wise multiplication. The “+1” operation is a residual identity mapping driven by [27, 47] that helps the network learn more robust attention maps by avoiding exploding or vanishes gradients (possibly caused by continuous layer-by-layer multiplication). *f*_*m*_(*i*) is learned in a self-supervised way through back propagation. Multiple attention modules are cascaded to extract high-expression feature maps more effectively. After that, we use global average pooling (GAP [48]) to replace the traditional fully connected layer in the convolutional neural network. The idea is to generate the corresponding feature map for each category in the classification task.

### 3.4. Information Interaction Module

In this section, we design a new method for information interaction between different task branches. In the auxiliary diagnosis task of myocardial infarction based on hand diagnosis of traditional Chinese medicine, we believe that even though specific branches of attention for different tasks focus on a certain part of the hand for feature extraction, each branch of attention for different tasks still has information that is beneficial to other branches of attention. Therefore, we build an information interaction module (IIM), through which the features of the same level in different attention modules of the attention branches of two specific tasks are fused.

We want the IIM module to capture more information that is useful for the specific task, rather than allowing specific task branches to fit freely without any interaction of information. Therefore, the IIM module alternately uses the output features of the attention modules of the two tasks as the main information and reference information. Firstly, the reference information features are given certain weight; then, they are interacted with the main information features. In this method, features with the same spatial resolution from different task branches are connected and dimensionality reduction is performed. This is conducive to cross-channel information interaction and helps the model to extract more distinctive features.

As shown in Figure 4, the output of the IIM module is mainly divided into two parts IIM_M_^*i*^ and IIM_P_^*i*^ (*i* represents the information interaction between the *i*-th attention module in the attention branch of two tasks). They represent the information interaction when different task branches are used as the main information and reference information, respectively. In particular, *F*_M,P_^*i*^ ∈ ℝ^*H*×*W*×*C*^ (*H*, *W*, and *C* are the height, width, and channel number of the feature graph, respectively) is defined as the output feature of the *i*-th attention module in the attention branch corresponding to task M or task P. In IIM_M_^*i*^, task M is the main information and task P is the reference information. In IIM_P_^*i*^, task P is the main information and task M is the reference information. We define the weight of the reference information in IIM_M_^*i*^ as *λ*_1_ and the weight of the reference information in IIM_*P*_^*i*^ as *λ*_2_. As shown in equation (5), the output of the IIM module can be defined as

(5) $$\begin{array}{c} \left\{\begin{array}{c} {\text{IIM}}_{\text{M}}^{i}=T_{1\times 1}\left(F_{\text{M}}^{i}⊕\lambda_{1}F_{\text{M}}^{i}\right),i\geq 1\\ {\text{IIM}}_{\text{P}}^{i}=T_{1\times 1}\left(F_{\text{P}}^{i}⊕\lambda_{2}F_{\text{P}}^{i}\right),i\geq 1 \end{array}\right\}. \end{array}$$

Here, *T*_1×1_ represents the convolution layer with the regularization and the convolution kernel of 1 × 1, and the stride is 1. It is worth noting that we use the 1 × 1 convolution layer because the 1 × 1 convolution kernel is able to perform calculations based on channels only, rather than fusing features of different spatial locations or changing the spatial size of features. In this way, the information interaction between channels is realized as well as dimension reduction. We also used batch normalization to enable stable learning. We train the IIM by backpropagating the task-specific losses and the *l*_2_ weight decay loss on the 1 × 1 convolutional weights.

### 3.5. Objective Function

Two of our tasks (task M, task P) were classified tasks. Therefore, the softmax function is used in the last layers of the two attention branches to predict the palmar thenar detection task (task P) and the metacarpophalangeal joint detection task (task M). As shown in equation (6), the cross-entropy loss of the palmar thenar detection task is expressed as

(6) $$\begin{array}{c} L_{t}=-\left[y^{t}\cdot \log\left(p^{t}\right)+\left(1-y^{t}\right)\cdot \log\left(1-p^{t}\right)\right], \end{array}$$

where *p*^*t*^ is the output of the model and *y*^*t*^ is the true label of the patient. For the loss of the metacarpophalangeal joint detection task, as shown in equation (7), cross-entropy loss is also adopted and expressed as

(7) $$\begin{array}{c} L_{k}=-\left[y^{k}\cdot \log\left(p^{k}\right)+\left(1-y^{k}\right)\cdot \log\left(1-p^{k}\right)\right], \end{array}$$

where *y*^*k*^ is the output of the model and *y*^*k*^ is the true label of the patient. Finally, we define the total loss function *L*_total_ as shown in

(8) $$\begin{array}{c} L_{\text{total}}\left(\sigma_{h},\sigma_{k}\right)=\frac{1}{2\sigma_{h}^{2}}L_{h}+\frac{1}{2\sigma_{k}^{2}}L_{k}+\log\sigma_{h}^{2}+\log\sigma_{k}^{2}. \end{array}$$

Inspired by [49], we adopt the method of uncertain weight to set task weight. *σ*_*h*_ and *σ*_*k*_ are learnable observation noise parameters.

## 4. Results

We introduced the dataset used for training and verification in Section 4.1. In Section 4.2, we introduced some implementation details in the experiment. In Section 4.3, we test the performance of our proposed method compared with the mainstream classification network. In addition, we also select several baseline networks and use comparative experiments to explain why other networks are not selected as the shared network for common feature extraction. In Section 4.4, we conducted some ablation experiments to verify the effectiveness of modules we proposed.

### 4.1. Dataset

In this work, we used a dataset containing cases of AMI patients from a cooperative Chinese medicine company. The dataset collected 2414 high-resolution hand images of 342 anonymous AMI patients, with labeled information by physicians with 20 years of rich experience in TCM diagnosis and treatment. In order to avoid the influence of light, angle, and other redundant factors, all image data are collected with professional equipment. However, for this study, we excluded images based on certain criteria: (1) images of severe peeling of the hand (*n* = 122), (2) images with scars in the palm area (*n* = 98), and (3) the palm that does not unfold naturally for various reasons or has more fingers and less fingers (*n* = 35). Because our research is a four-classification problem for two tasks, there were 570 images of palmar thenar hypertrophy with metacarpophalangeal joint swelling, 530 images of palmar thenar hypertrophy without metacarpophalangeal joint swelling, 522 images of metacarpophalangeal joint swelling without palmar thenar hypertrophy, and 537 images of both palmar thenar and metacarpophalangeal joint normal. In the end, 2414 tagged hand images were obtained from 301 patients (182 males and 119 females). We used 1931 for training and 483 for verification.

### 4.2. Implementation Details

All the experiments were conducted on a workstation with Ubuntu 18.04 LTS, Intel(R) Xeon(R) W-2102 CPU, and a NVIDIA TITAN XP GPU. We implemented MTIALM on the basis of PyTorch. We used the minibatch Adam optimizer (the basic learning rate is 0.01, beta_1_ is 0.9, beta_2_ is 0.999, epsilon is none, decay is 0, and batch size is 32) and set the maximum number of epoch to 500. In order to obtain better model performance, as shown in equation (9), we adopted the following learning rate variation scheme:

(9) $$\begin{array}{c} l\left(s\right)\left\{\begin{array}{c} l\left(0\right),0\leq s\leq 100\\ l\left(0\right)*0.5,100<s\leq 150\\ l\left(0\right)*0.1,150<s\leq 250\\ l\left(0\right)*0.01,250<s\leq 400\\ l\left(0\right)*0.001,400<s\leq 500 \end{array}\right\}, \end{array}$$

where *s* is the number of iterations and the initial learning rate *l*(0) is 0.01. During the training process, the model with the minimum total loss is saved to the validation set for validation on the test set. In order to avoid the slight imbalance of our dataset and overfitting of the model, as shown in equations (10) through (13), we evaluated the performance through accuracy, specificity, sensitivity, area under the receiver operator curve (AUC) [50], and *F*1-score. Their mathematical definition is as follows:

(10) $$\begin{array}{c} \text{Accuracy}=\frac{\text{TP}+\text{TN}}{\text{TP}+\text{FP}+\text{TN}+\text{FN}}, \end{array}$$

(11) $$\begin{array}{c} \text{Sensitivity}=\frac{\text{TP}}{\text{TP}+\text{FN}}, \end{array}$$

(12) $$\begin{array}{c} \text{Specificity}=\frac{\text{TN}}{\text{TN}+\text{FP}}, \end{array}$$

(13) $$\begin{array}{c} F1‐\text{score}=\frac{2\text{TP}}{2\text{TP}+\text{FN}+\text{FP}}, \end{array}$$

where TP represents the positive sample predicted by the model as a positive class, TN represents a negative sample predicted by the model as a negative class, FP represents a negative sample predicted by the model as a positive class, and FN represents a positive sample predicted by the model as a negative class.

### 4.3. Contrast Experiment

#### 4.3.1. Comparison of Classification Performance

At present, we have not found a similar study of TCM hand diagnosis based on traditional images. Therefore, in order to verify the performance of the proposed model, we apply several mainstream classification networks to our task and count the performance indicators of these methods.  Table 1 shows the performance comparison between the proposed MTIALM and several other classification networks in terms of accuracy, sensitivity, specificity, and *F*-score. In this comparison, our MTIALM outperformed all other methods in the task of detecting palmar thenar hypertrophy and metacarpophalangeal joint swelling based on traditional images. As shown in Figure 5, our method can achieve more than 83% accuracy in both tasks, which is about 4% higher than the best performance of ResNet-50 in other networks. We have performed a formal statistical analysis of the performance results of the model using uncorrected Dunn's test. We have performed a formal statistical analysis of the performance results of the model using uncorrected Dunn's test. We conducted comparative experiments on the training running time of different methods, as shown in Table 2. The experimental results show that compared with other methods, our method does not have much difference in running time with other methods while ensuring accuracy. In addition, we plotted the specificity and sensitivity of different models in Figures 6 and 7. They can show the stability and robustness of our MTIALM in the task of detecting palmar thenar hypertrophy and metacarpophalangeal joint swelling from different angles.

#### 4.3.2. Analysis of Baseline Shared Networks

In order to verify the effectiveness of choosing ResNet-18 as the shared network in our model, we calculate the performance indicators of different methods as the shared network.  Table 3 shows the comparison of accuracy, sensitivity, specificity, and *F*-score between the ResNet-18 used as the shared network and other networks (ResNet-50, VGG16, InceptionV3, MobileNet, etc.) used as the shared network. Since we use weights pretrained on the ImageNet dataset for transfer learning, we also use this approach for different baseline networks in the comparative experiment of common feature baseline networks. In this comparison, the results showed that the ResNet-18 we selected as the shared network was superior to other baseline networks. In the task of detecting palmar thenar hypertrophy, the accuracy was 82.23%, the sensitivity was 83.20%, the specificity was 78.38%, and the AUC was 84.47%. In the task of detecting metacarpophalangeal joint swelling, the accuracy was 84.46%, the sensitivity was 86.35%, the specificity was 79.47%, and the AUC was 85.39%.

### 4.4. Ablation Experiments

In this section, in order to further evaluate the effectiveness of the proposed specific task branch and the information interaction module (IIM module), we conducted several ablation experiments. Under the same training settings and the same dataset, we verified the performance of the modules mentioned in MTIALM, respectively, and evaluated them all according to the above indicators.

#### 4.4.1. Analysis of Attention Modules

In order to quantify the effectiveness of task-specific attention branch networks in the proposed method, we only used the shared network as the feature extraction method for the two tasks (OSN) and classified it. That is to say, we used ResNet-18 as the network of two tasks to independently detect metacarpophalangeal joint swelling and detect palmar thenar hypertrophy. As shown in Table 4, when the shared network is only used as the feature extraction network for each task, the performance of this method (OSN) is far lower than that of our method in each evaluation index.

In addition, in order to further verify the effectiveness of cascading attention modules, we combined the corresponding attention modules at different levels in the shared network and finally conducted 15 groups of experiments (including 4 sets of One-AM, 6 sets of Two-AM, 4 sets of Three-AM, and our proposed specific attention module). In order to solve the channel and image size matching problems during the ablation experiment, we used linear interpolation to achieve the unification of image size and 1 × 1 convolution to achieve the unification of image channels. For the combination of attention modules, as shown in Table 5, using only one attention module (One-AM), regardless of which layer of the shared network output is used as the input of the task-specific attention module, the result will result in the lowest performance (task M: the minimum accuracy was 51.24%, the minimum sensitivity was 53.45%, and the minimum specificity was 49.36%; task P: the minimum accuracy was 50.75%, the minimum sensitivity was 52.61%, and the minimum specificity was 50.13%). Using two task-specific attention modules (Two-AM) improves performance compared to using One-AM but is still not satisfactory. The reason for our analysis is that the two attention modules may still not be able to extract the distinguishing features well. For example, only low-dimensional features (1, 2 combination) or only high-dimensional features (3, 4 combination) cannot make the attention module play a real role. However, between the combination of low-dimensional features and high-dimensional features (1, 4 or other combinations), low-dimensional features need several times of subsampling before they can interact with high-dimensional features, which will lose too much information in this process.

In contrast, we found that four-task-specific attention module (MTIALM) cascades were most effective, and the accuracy, sensitivity, and specificity of metacarpophalangeal joint swelling task detection were 81.92%, 83.47%, and 79.93%, respectively. The accuracy, sensitivity, and specificity of the palmar thenar hypertrophy task were 82.46%, 84.11%, and 80.33%, respectively. By taking the layered features of the shared network as input to the attention modules for each specific task and cascading the attention modules layer by layer, the model can focus more on the most distinctive features. Therefore, we believe that task-specific attention branches formed by cascading attention modules are effective.

#### 4.4.2. Analysis of the Information Interaction Module

In order to demonstrate the advantages in the information interaction module (IIM), we compare the performance of our proposed model (MTIALM) with the model without the IIM module. To simplify, we validated the IIM module only on the basis of the best performance cascading four task-specific attention modules (MTIALM). The experimental results are shown in Table 6, which indicates that the accuracy of the model is significantly reduced after the deletion of the IIM module. As shown in Figures 8 and 9, we further illustrate the differences between MTIALM and noIIM-MTIALM in terms of performance and prevention of overfitting. In noIIM-MTIALM, the accuracy, sensitivity, and specificity of task M were 79.10%, 78.26%, and 83.33%, respectively, and those of task P were 80.64%, 79.51%, and 83.27%, respectively. These evaluation indexes were significantly lower than those of MTIALM. This means that the IIM module can learn more effective features through further interaction between features of different task branches by giving a certain weight to features of different branches. We hope that the IIM module can further help the task-specific attention branch network to act as a guide to help different tasks in the model focus on different areas, thus further extracting distinctive features.

For the setting of superparameters *λ*_1_ and *λ*_2_, we set the values of different superparameters, so as to determine the optimal scheme of information interaction between two task branches. Since there are two independent information interaction channels in the IIM module, there is no direct connection between the channels. Therefore, we separately verify the optimal values of *λ*_1_ and *λ*_2_. We first set *λ*_1_ in IIM_1_ to 0 and set five values (0.2, 0.4, 0.6, 0.8, and 1) for *λ*_2_ in IIM_2_ to verify the performance, respectively .After that, *λ*_2_ in IIM_2_ was set to 0 and *λ*_1_ in IIM_1_ was set to 5 values (0.2, 0.4, 0.6, 0.8, and 1) for experimental verification of performance. As shown in Table 7, we found that when *λ*_1_ and *λ*_2_ were 0.2 and 0.4, respectively, the performance of the model was the highest. It is worth noting that we did not choose 0 when we chose the value of *λ*, because when the value of *λ* is 0, it is equivalent to no information interaction between the two features, which means no IIM block is used. Therefore, we use 0.2 and 0.4 as the optimal values for *λ*_1_ and *λ*_2_.

In addition, in order to prove that the two tasks can promote each other in the process of model training, we remove the attention branches of two specific tasks, respectively, and observe the performance changes of the single task and multitask. The results are shown in Table 8. When the task branch for detecting palmar thenar hypertrophy was removed, the accuracy, sensitivity, and specificity of the task branch for detecting metacarpophalangeal joint swelling were 81.63%, 79.25%, and 82.77%, respectively. When the task branch of detecting metacarpophalangeal joint swelling was removed and only the task branch of detecting palmar thenar hypertrophy was retained, the accuracy, sensitivity, and specificity of detecting palmar thenar hypertrophy were 81.33%, 79.98%, and 83.30%, respectively. When the two tasks were performed simultaneously and the IIM module was added, the experimental results showed that the accuracy of both tasks was significantly improved. This further indicates that there are still some features between the two tasks that are conducive to improving the overall performance, and the IIM module we proposed can extract these features in the model training process.

## 5. Discussion

### 5.1. Visualization of the Deep Model

In order to further verify that the multitask attention model proposed by us has learned different features, we applied the gradient-weighted class activation mapping (Grad-CAM [51]) on the model. The visual result is shown in Figure 10. The brightness of part of the CAM image can indicate the extent to which the region is activated in the input image. The higher the brightness of a region, the more helpful it is for the model to predict the current task. The CAM image (Figures 10(a)–10(d)) is the task of predicting metacarpophalangeal joints. It can be seen that most of the high-activation areas show the metacarpophalangeal joint and surrounding areas of the hand. The CAM image (Figures 10(e)–10(h)) is the task of predicting palmar thenar hypertrophy, in which the high-activation areas exist in the surrounding area of the palmar thenar. These indicate that our method can better enable each task branch to focus on a specific area for learning, which is in line with the diagnostic methods of the related fields of traditional Chinese medicine hand diagnosis.

### 5.2. Research Limitation

Research limitations exist in two ways. First of all, our data is collected with professional equipment, excluding the influence of light, background, angle, and other factors. How to keep good performance without excluding the influence of these factors still needs further research. In addition, although our research has achieved good results, there is still room for improvement in the accuracy of prediction.

## 6. Conclusion

In this paper, we propose a new method based on a hand image to assist traditional Chinese medicine diagnosis of AMI, which can make good use of deep learning to assist traditional Chinese medicine to predict myocardial infarction. Our method is also a valuable attempt to combine traditional Chinese medicine hand diagnosis with artificial intelligence technology. Through a multitask interactive attention learning model (MTIALM), this method can detect the symptoms of two parts of the palm (metacarpophalangeal joints and palmar thenar) at the same time. Among them, in order to better realize the information interaction between the two tasks, we propose the new information interaction module (IIM). We used many evaluation indexes to carry out different experiments. From the experimental results, this method is more accurate than other traditional methods in two-task classification, and the model also has better stability and robustness. In the next research, we will combine more images to assist the prediction of myocardial infarction, in order to further improve the prediction performance.

## Figures and Tables

**Figure 1:** The framework of the proposed MTIALM. The input is the processed palm image, and then, the feature is extracted by the shared network (the shared network in the figure is ResNet-18). The shared network is connected to task-specific attention branch networks. There are two task-specific attention branches: the light blue branch (task M) is the task of detecting metacarpophalangeal joint swelling and the dark blue branch (task P) is the task of detecting palmar thenar hypertrophy. They each have their own set of attention modules. Its structure is shown in the second attention module. We connect the IIM module (grey) between the task-specific attention branches.

**Figure 2:** Explanation of the patch process. This figure shows how to cut a full-size palm image (a) into a patch image. Through four marked points (*X*_1_, *X*_2_, *Y*_1_, *Y*_2_), we can determine Δ*X* and Δ*Y*. Based on the determined *P*_size_, we can successfully extract the palm image without fingers (b).

**Figure 3:** Statistics of *P*_size_. The figure shows that the size of most palm areas is less than 460 pixels.

**Figure 4:** The framework of the proposed IIM. When the attention modules (task M and task P) of different tasks are input into the IIM, their feature maps are regarded as the main information and reference information, respectively. After the reference information is given a certain weight (blue translucent cube and orange translucent cube), it interacts with the main information. The useful channels of the final feature map are emphasized according to the depth of channel color.

**Figure 5:** Column bar graph plots of accuracy scores of different models.

**Figure 6:** Box-and-whisker plots of specificity scores of different models.

**Figure 7:** Box-and-whisker plots of sensitivity scores of different models.

**Figure 8:** Accuracy curve of two tasks under different methods.

**Figure 9:** Loss curve of two tasks under different methods.

**Figure 10:** Gradient-weighted class activation mapping images of the last convolution layer in MTIALM: (a–d) palm images of swollen metacarpophalangeal joints selected from four different patients; (e–h) images of palmar thenar hypertrophy selected from four different patients.

**Table 1:** Performance of different deep learning methods.

Methods	Task	Results (%)				
		Accuracy	Sensitivity	Specificity	*F*-score	*P* value
MTIALM	M	83.16 ± 2.11	84.71 ± 0.82	79.47 ± 4.16	81.25 ± 1.57	
	P	84.15 ± 3.07	85.79 ± 2.16	81.28 ± 2.72	82.91 ± 2.28	
ResNet-50	M	79.02 ± 2.35	83.49 ± 2.23	73.18 ± 5.34	80.36 ± 1.23	0.0204
	P	79.64 ± 4.03	84.02 ± 1.63	75.57 ± 4.19	82.33 ± 0.77	0.0301
DenseNet121	M	78.63 ± 0.36	80.42 ± 3.46	74.91 ± 1.40	74.12 ± 0.49	<0.001
	P	79.19 ± 2.31	83.06 ± 2.08	76.81 ± 2.48	75.63 ± 0.92	<0.001
VGG16	M	66.56 ± 1.24	67.81 ± 2.42	64.49 ± 3.32	65.94 ± 1.22	<0.001
	P	71.01 ± 0.48	73.44 ± 1.63	69.38 ± 1.71	68.71 ± 0.89	<0.001
AlexNet	M	63.01 ± 2.15	64.09 ± 2.20	60.29 ± 2.08	60.33 ± 1.87	<0.001
	P	65.29 ± 1.01	69.24 ± 1.01	62.51 ± 1.33	63.59 ± 3.01	<0.001
InceptionV3	M	66.28 ± 2.27	69.25 ± 3.31	65.38 ± 1.17	63.97 ± 4.11	<0.001
	P	68.25 ± 1.77	69.58 ± 1.83	65.26 ± 1.91	65.29 ± 3.18	<0.001
MobileNet	M	72.37 ± 4.13	75.39 ± 3.67	71.33 ± 3.47	71.86 ± 2.92	<0.001
	P	73.02 ± 2.19	78.26 ± 2.21	69.28 ± 2.63	71.88 ± 1.45	<0.001

**Table 2:** Comparison of training running time of different methods.

Methods	MTIALM	ResNet-50	DenseNet121	VGG16	AlexNet	InceptionV3	MobileNet
Time (min/epoch)	0.45	0.43	0.47	0.52	0.24	0.37	0.25

**Table 3:** Performance of different shared networks.

Shared network	Task	Results (%)			
		Accuracy	Sensitivity	Specificity	AUC
ResNet-18	M	82.23 ± 3.46	83.20 ± 1.13	78.38 ± 3.54	84.47 ± 0.32
	P	84.46 ± 4.31	86.35 ± 0.22	79.47 ± 2.72	85.39 ± 0.27
ResNet-34	M	79.37 ± 1.78	82.38 ± 1.01	75.24 ± 2.21	81.74 ± 0.44
	P	80.33 ± 2.81	83.81 ± 2.25	74.89 ± 3.41	83.09 ± 1.05
ResNet-50	M	82.03 ± 1.83	83.31 ± 0.77	78.37 ± 2.51	84.21 ± 1.13
	P	82.57 ± 1.23	84.06 ± 1.15	79.32 ± 3.18	84.33 ± 0.65
VGG16	M	67.73 ± 1.87	71.34 ± 3.03	64.25 ± 5.17	69.24 ± 1.03
	P	71.56 ± 0.35	72.05 ± 2.76	67.62 ± 6.38	73.87 ± 0.93
AlexNet	M	63.46 ± 3.51	66.40 ± 3.16	60.74 ± 3.92	65.37 ± 2.16
	P	68.98 ± 2.89	70.28 ± 4.35	63.68 ± 5.03	70.45 ± 0.86
InceptionV3	M	68.45 ± 3.24	70.33 ± 3.07	62.76 ± 4.91	69.57 ± 0.62
	P	69.71 ± 1.87	72.48 ± 2.89	65.03 ± 2.38	71.22 ± 1.19
MobileNet	M	74.36 ± 3.10	77.23 ± 2.17	69.71 ± 4.17	76.35 ± 0.27
	P	74.76 ± 2.66	76.25 ± 1.79	70.29 ± 3.02	78.25 ± 0.46

**Table 4:** Evaluation result of the models with or without attention modules.

Models	Task	Result (%)				
		Accuracy	Sensitivity	Specificity	AUC	*F*-score
MTIALM	M	82.43	81.05	84.27	82.91	81.35
	P	83.03	81.33	84.65	84.13	81.65
OSN	M	78.35	75.26	79.16	79.41	79.37
	P	78.86	76.83	80.01	79.80	80.50

**Table 5:** Evaluation result of different attention module combinations.

Models	Component				Task	Result (%)			
	1	2	3	4		Accuracy	Sensitivity	Specificity	AUC
One-AM-1	√				M	51.24	53.45	49.36	52.39
					P	50.75	52.61	50.13	52.11
One-AM-2		√			M	51.78	54.14	51.01	54.21
					P	53.16	56.73	51.84	55.59
One-AM-3			√		M	57.28	59.31	53.82	58.37
					P	54.53	59.46	52.44	58.84
One-AM-4				√	M	62.21	64.57	58.30	64.73
					P	62.55	63.79	60.15	65.03
Two-AM-1	√	√			M	56.41	59.73	53.51	57.32
					P	54.89	56.56	51.74	56.56
Two-AM-2	√		√		M	62.81	65.82	58.66	64.39
					P	62.17	66.15	60.59	62.95
Two-AM-3	√			√	M	66.15	69.81	62.54	68.26
					P	65.23	67.48	62.05	68.47
Two-AM-4		√	√		M	62.79	65.22	59.57	65.01
					P	61.97	63.98	57.18	64.56
Two-AM-5		√		√	M	67.09	70.02	65.91	71.63
					P	65.77	67.57	61.10	69.05
Two-AM-6			√	√	M	73.80	74.46	67.09	75.79
					P	70.19	73.11	64.96	74.14
Three-AM-1	√	√	√		M	76.21	78.40	69.38	79.52
					P	74.26	77.03	69.65	77.31
Three-AM-2	√	√		√	M	73.46	77.73	71.09	76.37
					P	73.10	74.95	70.33	73.96
Three-AM-3	√		√	√	M	72.59	74.30	68.72	75.93
					P	73.33	76.24	70.65	77.01
Three-AM-4		√	√	√	M	76.68	80.33	75.03	79.36
					P	78.21	82.06	74.29	80.65
Four-AM (ours)	√	√	√	√	M	81.92	83.47	79.93	82.30
					P	82.46	84.11	80.33	83.27

**Table 6:** Evaluation results of the models with or without the CA block.

Models	Task	Result (%)				
		Accuracy	Sensitivity	Specificity	AUC	*F*-score
MTIALM	M	82.23	80.63	83.73	84.28	81.33
	P	83.03	80.75	84.66	84.71	81.75
noIIM-MTIALM	M	79.10	78.26	83.33	83.89	78.23
	P	80.64	79.51	83.27	83.65	80.16

**Table 7:** Evaluation results of two different weight combinations in the IIM module.

(*λ*_1_, *λ*_2_)	Task	Result (%)				
		Accuracy	Sensitivity	Specificity	AUC	*F*-score
(0, 0.2)	M	81.02	79.23	83.21	82.25	79.39
	P	80.37	78.16	81.91	82.01	79.31
(0, 0.4)	M	82.71	80.85	84.79	83.03	81.45
	P	82.26	81.11	84.63	82.98	81.27
(0, 0.6)	M	82.39	80.16	83.33	83.92	81.02
	P	81.72	81.21	82.70	83.54	81.25
(0, 0.8)	M	80.35	78.24	81.26	82.22	78.14
	P	80.54	78.93	82.38	82.83	80.03
(0, 1)	M	79.29	78.45	80.35	81.44	77.76
	P	80.06	78.82	82.96	82.07	78.31
(0.2, 0)	M	82.84	80.02	83.29	83.03	80.15
	P	83.45	80.89	84.67	84.41	81.73
(0.4, 0)	M	81.10	79.24	83.25	82.74	79.31
	P	82.26	80.23	83.33	83.67	81.20
(0.6, 0)	M	80.43	78.85	81.01	82.03	78.26
	P	81.93	79.64	80.40	82.39	79.33
(0.8, 0)	M	80.22	78.65	81.23	81.42	78.35
	P	80.47	78.38	82.17	81.89	78.94
(1, 0)	M	78.91	75.42	80.52	80.30	77.43
	P	79.09	78.51	81.33	81.35	78.41

**Table 8:** Evaluation results of the single task and multitask in the model.

Models	Task	Result (%)				
		Accuracy	Sensitivity	Specificity	AUC	*F*-score
MTIALM	M	82.06	80.20	83.39	83.86	81.27
	P	82.96	81.07	84.35	84.39	81.24
MTIALM-no M	P	81.33	79.98	83.30	83.62	80.04
MTIALM-no P	M	81.63	79.25	82.77	83.20	80.51

## Data Availability

The datasets of images used to support the findings of this study are available from the corresponding author upon request.

## References

[1] Li J., Zhang B., Lu G., You J., Zhang D. (2019). Body surface feature-based multi-modal learning for diabetes mellitus detection. *Information Sciences*.

[2] Guzmán J. C., Miramontes I., Melin P., Prado-Arechiga G. (2019). Optimal genetic design of type-1 and interval type-2 fuzzy systems for blood pressure level classification. *Axioms*.

[3] Lin S., Li Z., Fu B. (2020). Feasibility of using deep learning to detect coronary artery disease based on facial photo. *European Heart Journal*.

[4] Zhang Q., Zhou J., Zhang B., Wu E., Cun X. (2021). DsNet: dual stack network for detecting diabetes mellitus and chronic kidney disease. *Information Sciences*.

[5] Su W., Xu Z. Y., Wang Z. Q., Xu J. T. (2011). Objectified study on tongue images of patients with lung cancer of different syndromes. *Chinese Journal of Integrative Medicine*.

[6] Yan K., Zhang D., Wu D., Wei H., Lu G. (2014). Design of a breath analysis system for diabetes screening and blood glucose level prediction. *IEEE Transactions on Biomedical Engineering*.

[7] Peng Wang, Wangmeng Zuo, Zhang D. (2014). A compound pressure signal acquisition system for multichannel wrist pulse signal analysis. *IEEE Transactions on Instrumentation and Measurement*.

[8] Kirschbaum B. (2000). Atlas of Chinese tongue diagnosis. *Eastland Pr*.

[9] Yan K., Kou L., Zhang D. (2018). Learning domain-invariant subspace using domain features and Independence maximization. *IEEE Transactions on Cybernetics*.

[10] Li B., Huang Q., Lu Y., Chen S., Liang R., Wang Z., Zhang D. (2007). A method of classifying tongue colors for traditional Chinese medicine diagnosis based on the CIELAB color space. *Medical Biometrics. ICMB 2008*.

[11] Zhang D., Pang B., Li N., Wang K., Zhang H. (2005). Computerized diagnosis from tongue appearance using quantitative feature classification. *The American Journal of Chinese Medicine*.

[12] Wang D., Zhang D., Lu G. (2017). Generalized feature extraction for wrist pulse analysis: from 1-D time series to 2-D matrix. *IEEE Journal of Biomedical and Health Informatics*.

[13] Zhang Y., Rong L., Wang Z. (2005). Analysis of the color characteristics of tongue digital images of 884 cases from the persons received a general physical examination. *Journal of Beijing University of Traditional Chinese Medicine*.

[14] Li C.-h., Yuen P. C. (2002). Tongue image matching using color content. *Pattern Recognition*.

[15] Zhang D., Zhang H., Zhang B. (2017). Tongue shape classification by geometric features. *Tongue Image Analysis*.

[16] Xingzheng Wang, Zhang B., Zhimin Yang, Haoqian Wang, Zhang D. (2013). Statistical analysis of tongue images for feature extraction and diagnostics. *IEEE Transactions on Image Processing*.

[17] Kim B., Lee S., Cho D., Oh S. A proposal of heart diseases diagnosis method using analysis of face color.

[18] Liu M., Guo Z., Zhang D. (2007). Hepatitis diagnosis using facial color image. *Medical Biometrics. ICMB 2008*.

[19] Baloglu U. B., Talo M., Yildirim O., Tan R. S., Acharya U. R. (2019). Classification of myocardial infarction with multi-lead ECG signals and deep CNN. *Pattern Recognition Letters*.

[20] Zeng W., Yuan J., Yuan C., Wang Q., Liu F., Wang Y. (2020). Classification of myocardial infarction based on hybrid feature extraction and artificial intelligence tools by adopting tunable-Q wavelet transform (TQWT), variational mode decomposition (VMD) and neural networks. *Artificial Intelligence in Medicine*.

[21] Chen M., Fang L., Zhuang Q., Liu H. (2019). Deep learning assessment of myocardial infarction from MR image sequences. *IEEE Access*.

[22] Acharya U. R., Fujita H., Oh S. L., Hagiwara Y., Tan J. H., Adam M. (2017). Application of deep convolutional neural network for automated detection of myocardial infarction using ECG signals. *Information Sciences*.

[23] Jafarian K., Vahdat V., Salehi S., Mobin M. (2020). Automating detection and localization of myocardial infarction using shallow and end-to-end deep neural networks. *Applied Soft Computing*.

[24] Xu K., Ba J. L., Kiros R. Show, attend and tell: neural image caption generation with visual attention.

[25] Hu J., Shen L., Albanie S., Sun G., Wu E. (2020). Squeeze-and-excitation networks. *IEEE Transactions on Pattern Analysis and Machine Intelligence*.

[26] Li X., Wang W., Hu X., Yang J. Selective kernel networks.

[27] He K., Zhang X., Ren S., Sun J., Leibe B., Matas J., Sebe N., Welling M. Identity mappings in deep residual networks. *Computer Vision – ECCV 2016. ECCV 2016*.

[28] Park J., Woo S., Lee J.-Y., Kweon I.-S. (2018). *BAM: Bottleneck Attention Module*.

[29] Woo S., Park J., Lee J. Y., Kweon I. S., Ferrari V., Hebert M., Sminchisescu C., Weiss Y. CBAM: convolutional block attention module. *Computer Vision – ECCV 2018. ECCV 2018*.

[30] Fu J., Liu J., Tian H. Dual attention network for scene segmentation.

[31] Cao Y., Xu J., Lin S., Wei F., Hu H. GCNet: non-local networks meet squeeze-excitation networks and beyond.

[32] Xu D., Ouyang W., Wang X., Sebe N. PAD-Net: multi-tasks guided prediction-and-distillation network for simultaneous depth estimation and scene parsing.

[33] He K., Gkioxari G., Dollár P., Girshick R. Mask R-CNN.

[34] Eigen D., Fergus R. Predicting depth, surface normals and semantic labels with a common multi-scale convolutional architecture.

[35] Kokkinos I. UberNet: training a universal convolutional neural network for low-, mid-, and high-level vision using diverse datasets and limited memory.

[36] Misra I., Shrivastava A., Gupta A., Hebert M. Cross-stitch networks for multi-task learning.

[37] Maninis K., Radosavovic I., Kokkinos I. Attentive single-tasking of multiple tasks.

[38] Vandenhende S., Georgoulis S., Van Gool L., Vedaldi A., Bischof H., Brox T., Frahm J. M. (2020). MTI-Net: multi-scale task interaction networks for multi-task learning. *Computer Vision – ECCV 2020. ECCV 2020*.

[39] Teichmann M., Weber M., Zöllner M., Cipolla R., Urtasun R. MultiNet: real-time joint semantic reasoning for autonomous driving.

[40] Zhang Z., Cui Z., Xu C., Jie Z., Li X., Yang J., Ferrari V., Hebert M., Sminchisescu C., Weiss Y. (2018). Joint task-recursive learning for semantic segmentation and depth estimation. *Computer Vision – ECCV 2018. ECCV 2018*.

[41] Thung K.-H., Wee C.-Y. (2018). A brief review on multi-task learning. *Multimedia Tools and Applications*.

[42] Vandenhende S., Georgoulis S., Proesmans M., Dai D., Van Gool L. Revisiting multi-task learning in the deep learning era.

[43] Yildirim P., Birant K., Birant D. (2020). Multitask-based association rule mining. *Turkish Journal of Electrical Engineering and Computer Sciences*.

[44] He K., Zhang X., Ren S., Sun J. Deep residual learning for image recognition.

[45] Deng J., Dong W., Socher R., Li L., Li K., Fei-Fei L. ImageNet: a large-scale hierarchical image database.

[46] Ioffe S., Szegedy C. Batch normalization: accelerating deep network training by reducing internal covariate shift.

[47] Wang F., Jiang M., Qian C. Residual attention network for image classification.

[48] Lin M., Chen Q., Yan S. (2014). Network in network. *2nd International Conference on Learning Representations, ICLR 2014 - Conference Track Proceedings. International Conference on Learning Representations, ICLR*.

[49] Cipolla R., Gal Y., Kendall A. Multi-task learning using uncertainty to weigh losses for scene geometry and semantics.

[50] Jin Huang, Ling C. X. (2005). Using AUC and accuracy in evaluating learning algorithms. *IEEE Transactions on Knowledge and Data Engineering*.

[51] Selvaraju R. R., Cogswell M., Das A., Vedantam R., Parikh D., Batra D. Grad-CAM: visual explanations from deep networks via gradient-based localization.

